# A Meta-Analysis of Robotic Surgery in Endometrial Cancer: Comparison with Laparoscopy and Laparotomy

**DOI:** 10.1155/2020/2503753

**Published:** 2020-01-21

**Authors:** Jia Wang, Xiaomao Li, Haotian Wu, Yu Zhang, Fei Wang

**Affiliations:** The Third Affiliated Hospital of Sun Yat-sen University, Guangzhou 510630, China

## Abstract

**Background:**

The safety and effectiveness of robotic surgery are evaluated by comparing perioperative outcomes with laparoscopy and laparotomy in endometrial cancer.

**Method:**

PubMed, MEDLINE, Embase, Cochrane, and other databases were searched for eligible studies up to April 2019. Studies that compared robotic surgery with laparoscopy or laparotomy in surgical staging of endometrial cancer were included. The pooled odds ratio and weighted mean difference were calculated using a random-effects or a fixed-effects model to summarize the results.

**Results:**

Twenty-seven articles were ultimately included, with one randomized controlled trial and 26 observational studies. A total of 6568 patients were included. Meta-analysis showed that robotic surgery had less estimated blood loss (*P* < 0.001), blood transfusion (*P* = 0.04), intraoperative complications (*P* = 0.001), and conversion to open surgery (*P* = 0.001), and a shorter hospital stay (*P* = 0.001), but had a longer operation time (*P* = 0.04) in surgical staging of endometrial cancer compared with laparoscopy. There were no significant differences in postoperative complications, the total number of lymph nodes harvested, the number of pelvic lymph nodes harvested, and the number of para-aortic lymph nodes harvested between techniques. Robotic surgery had a longer operation time (*P* = 0.008), less estimated blood loss (*P* < 0.001), blood transfusion (*P* < 0.001), and postoperative complications (*P* < 0.001), and a shorter hospital stay (*P* < 0.001) compared with laparotomy. There were no significant differences in other variables between techniques.

**Conclusion:**

Robotic surgery is a safer surgical approach than laparoscopy and laparotomy in surgical staging of endometrial cancer, with less estimated blood loss, blood transfusion, and conversion, and the same number of lymph nodes harvested.

## 1. Introduction

Endometrial cancer is the fifth most common cancer in women worldwide. The incidence and death rates of endometrial cancer have increased in recent years, particularly in industrialized countries. Surgery is the major treatment for endometrial cancer, for cutting out tumors and providing a surgical stage, which can guide the choice of postoperative adjuvant treatment. At present, vaginal surgery, laparotomy (LT), laparoscopic surgery (LPS), and robotic surgery (RS) can be used to treat endometrial cancer. In 1993, Childers first proposed laparoscopy as an option for early-stage endometrial cancer. The largest randomized controlled trial (RCT) to compare LPS with LT is the GOG trial, LAP-2. This trial showed that patients who underwent LPS for endometrial cancer had improved short-term and survival outcomes compared with those who underwent LT [1, 2]. In January 1999, the Da Vinci robotic surgery system was developed, and it received initial clearance from the US Food and Drug Administration in 2005 for the gynecological field. In recent years, technology related to robots has improved. Currently, approximately 80% of patients undergo hysterectomy for cancer by robotic surgery in the USA [3]. However, the advantage of RS relative to LPS and LT in the treatment of endometrial cancer has not been determined. Therefore, in this study, we performed a meta-analysis to compare the perioperative outcome of different surgical approaches to evaluate the advantages of robotic surgery in the staging of endometrial cancer.

## 2. Methods

### 2.1. Study Search

We searched PubMed, Cochrane Libraries, MEDLINE, Embase, Ovid, Web of Science, and ScienceDirect up to April 2019. The search terms used a combination of keywords and MeSH terms as follows: “endometrial carcinoma,” “endometrial cancer,” “uterine cancer,” “robotic,” “laparoscopic,” “laparoscopy,” and “laparotomy.” Additional relevant references were searched for references of eligible articles. EndNote was used to merge retrieved citations and eliminate duplications. Gray literature and conference abstracts were not included in the search. The authors of this study carried out the search independently.

### 2.2. Outcome Measures

We compared the surgical effect not only between RS and LPS but also between RS and LT. The following perioperative outcomes were used: operation time (OT), estimated blood loss (EBL), intraoperative complications, postoperative complications, blood transfusion, conversion to laparotomy, total lymph nodes harvested (TLNH), the number of pelvic lymph nodes harvested (PLNH), the number of para-aortic lymph nodes harvested (PALNH), and hospital stay.

### 2.3. Inclusion and Exclusion Criteria

The inclusion criteria were as follows: (1) Studies needed to be published in English, and RCTs and prospective or retrospective observational studies were included. When the same institution reported more than one study, only the largest and most informative studies were included. (2) Patients who were diagnosed with endometrial cancer were included. (3) Interventions included comparison of RS (treatment arm) with LPS or LT (control arm) for the treatment of endometrial cancer. (4) At least one of the outcomes of interest was reported.

The exclusion criteria were as follows: (1) duplicate publications, case series, case reports, reviews, conference abstracts, editorials, and letters; (2) studies with patients who received radiation therapy or chemotherapy preoperation; (3) studies without appropriate data that could be extracted or calculated; and (4) series with less than 25 cases of RS were excluded to minimize potential learning curve bias [4, 5]. Two authors independently selected studies for inclusion, and differences were resolved by discussion.

### 2.4. Data Extraction and Quality Assessment

This meta-analysis was performed in accordance with meta-analysis of observational studies in epidemiology (MOOSE) guidelines [6]. Data extraction and quality assessment were carried out by J.W. and HT.W. using a prespecified data collection form. For continuous variables, the sample size, mean, and standard deviation (SD) were calculated. For dichotomous variables, the total number of patients in each group and the number of events were calculated. If studies reported the median rather than mean values, and range or interquartile range rather than SD, the mean and SD were estimated [7]. Additionally, we extracted characteristics of each study, including the first author's name, year, country of publication, number of research centers, study period, type of study, whether the surgeon was the same, and the participants' age and body mass index. Assessment of RCTs was according to the Cochrane Collaboration tool in the Cochrane Handbook [8]. Quality assessment of a nonrandomized controlled trial was assessed using the criteria developed by the Newcastle-Ottawa Scale (NOS) [9, 10]. This scale uses the semiquantification principle of the star rating system. The evaluation project consists of eight items, and studies with six or more stars were considered to be of much higher quality. Disagreements were resolved through discussion under supervision of a third reviewer (XM.L.).

### 2.5. Statistical Analysis

The data were analyzed by Review Manager 5.3 (RevMan 5.3, The Cochrane Collaboration, Oxford, UK). The weighted mean difference (WMD) and 95% confidence interval (CI) were used for summary variables for continuous outcomes, and the risk ratio (RR) and 95% CI were used for dichotomous variables. Heterogeneity of the studies was examined within two types of study design using Cochrane's *Q* test of heterogeneity and the *I*^2^ statistic, which provides the relative amount of variance of the summary effect due to between-study heterogeneity [8, 11]. When there was significant heterogeneity (*P* < 0.10, *I*^2^ ≥ 50%), we used the random-effects model. Otherwise, the fixed-effects model was used. Sensitivity analyses were used when potential clinical heterogeneity existed without statistical heterogeneity or there was a risk of bias associated with the quality [8]. These analyses were performed by omitting one study each time. Subgroup analyses were performed by omitting studies within the same category. Publication bias was evaluated by funnel plots. Begg's and Egger's tests were used to detect funnel plot asymmetry.

## 3. Results

### 3.1. Study Characteristics

Figure 1 shows the flow chart of the study selection process. The literature search extracted 11,585 articles from the database search and relevant references. Most of the articles were excluded after the first screening of the title and abstract. A total of 47 articles were read in full. Of these, we excluded 20 studies for the following reasons: one study was not published in English, 10 did not report the outcomes of interest, five did not meet the 25 robotic case limit threshold, two were duplicates, one was an abstract only, and one was not a comparison study. Finally, 27 studies [5, 12–37] were included in this analysis. A total of 6568 patients were identified: 2253 patients in the RS group, 1996 patients in the LPS group, and 2319 patients in the LT group.

More detailed information and the clinical characteristics of the included studies are shown in Table 1. The studies were published between 2008 and 2019. Fifteen studies were conducted in the United States, Italy, and Finland (two studies in each of these countries), and in Canada, Sweden, France, Spain, Taiwan, Korea, Thailand, and Singapore (one study in each country). One study was a RCT [27]. Twenty-six studies were observational studies, and 20 of these were retrospective and six were prospective. Among the studies, 12 compared RS, LPS, and LT, nine compared RS and LPS, and six compared RS and LT.

We performed quality assessment of observational studies with the NOS and the RCT with the Cochrane Handbook 5.1.0. The NOS scores of the 26 observational studies ranged from seven to nine stars; seven studies [5, 15, 17, 19, 22, 36, 37] had nine stars, 12 studies [12, 14, 20, 21, 23–26, 28, 30, 33, 34] had eight stars, and seven studies [13, 16, 18, 29, 31, 32, 35] had seven stars. The RCT and all of the observational studies were of high quality (Table S2).

### 3.2. Outcome

#### 3.2.1. RS vs. LPS

1. OT: twenty-one studies [5, 12–17, 21–23, 25–29, 32–37] reported the OT. The OT was significantly longer in the RS group than in the LPS group (WMD, 19.87; 95% CI, 0.60–39.15; *P* = 0.04; Figure 2)
2. EBL: nineteen studies [5, 12–17, 21–23, 25, 27–29, 31, 33, 35–37] reported the EBL. EBL appeared to be less in the RS group than in the LPS group, but this difference was not significant (WMD, -53.66; 95% CI, -74.86 to -32.47; *P* < 0.001; Figure 3)
3. Intraoperative complications: intraoperative complications included intestinal injury, bladder injury, vaginal laceration, intraoperative bleeding >500 ml, and inferior vena cava injury. Seventeen studies [5, 12–14, 16, 17, 21, 23, 25–29, 32–35] reported intraoperative complications. There were significantly fewer intraoperative complications in the RS group than in the LPS group (RR, 0.52; 95% CI, 0.35–0.77; *P* = 0.001; Figure S1)
4. Postoperative complications: postoperative complications included deep vein thrombosis, pulmonary embolism, intestinal obstruction, fever, vaginal cuff infection, pelvic abscess, wound infection, hernia, vaginal cuff cracking, and lymphedema. Thrombotic thrombosis was one of the most common postoperative complications. Sixteen studies [5, 12–17, 22, 23, 25–29, 34, 35] reported postoperative complications. There appeared to be fewer postoperative complications in the RS group than in the LPS group, but this was not significant (RR, 0.69; 95% CI, 0.76–1.20; *P* = 0.69; Figure S2)
5. Blood transfusion: thirteen studies [12–14, 16, 17, 21, 22, 26–29, 33, 34] reported blood transfusion. There was significantly less blood transfusion in the RS group than in the LPS group (RR, 0.65; 95% CI, 0.44–0.96; *P* = 0.03; Figure S3)
6. Conversion: fourteen studies [5, 13, 14, 16, 17, 21–23, 25–28, 33, 35] reported conversion. The rate of conversion was significantly lower in the RS group than in the LPS group (RR, 0.55; 95% CI, 0.38–0.81; *P* = 0.002; Figure S4)
7. TLNH: ten studies [5, 12–15, 22, 23, 27, 36, 37] reported the TLNH. There appeared to be more TLNH in the RS group than in the LPS group, but this difference was not significant (WMD, 0.73; 95% CI, -3.62 to 5.08; *P* = 0.74; Figure S5)
8. PLNH: ten studies [5, 13, 14, 16, 17, 21, 25, 26, 28, 33] reported the number of PLNH. There appeared to be a greater number of PLNH in the RS group than in the LPS group, but this difference was not significant (WMD, 0.72; 95% CI, -2.85 to 4.29; *P* = 0.69; Figure S6)
9. PALNH: ten studies [5, 13, 14, 16, 17, 21, 25, 26, 28, 33] reported the number of PALNH. There appeared to be a greater number of PALNH in the LPS group than in the RS group, but this difference was not significant (WMD, -0.09; 95% CI, -2.93 to 2.75; *P* = 0.95; Figure S7)
10. Hospital stay: twenty studies [5, 12–17, 21–23, 25–29, 32–35, 37] reported hospital stay. Hospital stay was significantly shorter in the RS group than in the LPS group (WMD, -0.35; 95% CI, -0.54 to -0.17; *P* = 0.0001; Figure S8)

#### 3.2.2. Robotic Surgery vs. Laparotomy

(1) OT: eighteen studies [12, 13, 15–20, 22, 24–26, 28–32, 35] reported the OT. The OT was significantly shorter in the LT group than in the RS group (WMD, 29.97; 95% CI, 7.60–50.35; *P* = 0.008; Figure 4)

(2) EBL: seventeen studies [12, 13, 15–20, 22, 24, 25, 28–32, 35] reported EBL. EBL was significantly less in the RS group than in the LT group (WMD, -147.02; 95% CI, -185.72 to -108.31; *P* < 0.00001; Figure 5)

(3) Intraoperative complications: fourteen studies [12, 13, 16, 17, 19, 20, 25, 26, 28–32, 35] reported intraoperative complications. There appeared to be fewer complications in the RS group than in the LT group (RR, 0.76; 95% CI, 0.53–1.10; *P* = 0.15; Figure S9). However, even though a large number of studies reported fewer complications in the RS group, this difference was not significant

(4) Postoperative complications: fifteen studies [12, 13, 15–17, 19, 20, 22, 25, 26, 28–31, 35] reported postoperative complications. There were significantly fewer complications in the RS group than in the LT group (RR, 0.41; 95% CI, 0.33–0.50; *P* < 0.00001; Figure S10)

(5) Blood transfusion: ten studies [12, 13, 16–18, 22, 26, 28, 29, 31] reported blood transfusion. There was significantly less blood transfusion in the RS group than in the LT group (RR, 0.22; 95% CI, 0.15–0.32; *P* < 0.00001; Figure S11)

(6) TLNH: seven studies [12, 13, 15, 18–20, 22] reported the TLNH. There appeared to be more TLNH in the RS group than in the LT group, but this difference was not significant (WMD, 3.30; 95% CI, 0.06–6.54; *P* = 0.05; Figure S12)

(7) PLNH: nine studies [13, 16–18, 24–26, 28, 30] reported the number of PLNH. There appeared to be more PLNH in the LT group than in the RS group, but this difference was not significant (WMD, -0.39; 95% CI, -3.10 to 2.32; *P* = 0.78; Figure S13)

(8) PALNH: eight studies [13, 16–18, 24–26, 28] reported the number of PALNH. There appeared to be more PALNH in the RS group than in the LT group, but this difference was not significant (WMD, 0.43; 95% CI, -1.58 to 2.45; *P* = 0.67; Figure S14)

(9) Hospital stay: eighteen studies [12, 13, 15–20, 22, 24–26, 28–32, 35] reported hospital stay. Hospital stay in the RS group was significantly shorter than that in the LT group (WMD, -2.76; 95% CI, -3.08 to -2.43; *P* < 0.00001; Figure S15)

#### 3.2.3. Publication Bias

Visual inspection of Begg's funnel plots of intraoperative complications showed that there was no obvious asymmetry, which indicated no evidence of publication bias among the studies for outcomes of intraoperative complication of RS versus LPS (Figure S16(a)) and RS versus LT (Figure S16(b)). The funnel plots of the other outcomes also showed no significant heterogeneity and no publication bias in this meta-analysis (figures not shown).

## 4. Discussion

In recent years, with the development of evidence-based medicine, a large number of meta-analyses based on RCTs have been used to guide clinical practice. However, some medical problems, with restriction of medical ethics, characteristics of the human body, or implementation of constraints, make performing a RCT difficult. In contrast to RCTs, observational studies have a greater risk of selection bias, but they comprise a large proportion of medical research and provide important information. Therefore, meta-analysis of observational studies remains important.

Endometrial cancer is the fifth most common cancer in women worldwide. Its development is related to many signaling pathways [38–40]. Surgery is the main treatment of endometrial cancer. Safe and effective treatment is important for prognosis of the disease and improved quality of life of the patients. In recent years, multiple methods have been developed to perform staging surgery for endometrial cancer. In the last decade, a few studies have compared perioperative outcomes of the three surgical approaches for endometrial cancer. Because the scale of the studies was small and the results varied, evidence to support the use of RS in endometrial cancer is still lacking. Therefore, this meta-analysis is aimed at verifying the potential advantages of RS and help the surgeon to understand the present status of robotic surgery in gynecology.

Safety is the most important consideration when a new surgical technique is developed. Intraoperative and postoperative complications, EBL, transfusion, and conversion are effective indicators for evaluating the safety of surgical techniques. Our study showed that RS has less EBL, a lower rate of complications, a lower rate of conversion, and shorter hospital stay in the staging of endometrial cancer compared with LPS and LT. These advantages of RS might be attributed to the following factors: (1) RS offers 3D visualization of the operative field, which allows better detection of large and small vessels to avoid unnecessary damage. (2) Wrist motion allows better dexterity and precision that can mimic freedom of the human hand. This can avoid mistakes and make suturing and complicated dissection easier. (3) RS decreases musculoskeletal fatigue in surgeons.

We found no significant difference in the OT between RS and LPS, but the time required for LPS was relatively shorter. The operation time of LT was significantly shorter than that of RS. Seror et al. [34] and Venkat et al. [37] reported that RS resulted in a longer time in the operating room and longer operation time compared with LPS (*P* = 0.003, *P* = 0.01; *P* < 0.001, *P* < 0.001, respectively). Seamon et al. [33] showed that RS has a significantly longer operating room to incision time than that of LPS (*P* = 0.009). Additionally, the skin incision to skin closure time in LPS was significantly longer than that of RS (*P* < 0.001). Jiménez Rodríguez et al. [41] pointed out that the preparation time of the Da Vinci robotic surgery system was longer than that of traditional LPS, but the real operation time was not significantly different between the two groups. Payne and Dauterive [42] also found that the installation and preparation times have become a disadvantage in robotic surgery.

Comprehensive lymphadenectomy is an important part of endometrial cancer staging. Complete lymphadenectomy should include pelvic lymph node resection and para-aortic lymph node resection. The number of lymph nodes that are removed might be the most important parameter for lymphadenectomy, and is also a measure of surgical quality [13]. Diaz-Feijoo et al. [43] compared the data of 100 consecutive cases of lymph node resection in RS and LPS. They showed that median lymph node resection in RS was greater than that in LPS (17 (10–31) vs. 14 (4–62), *P* < 0.05). Our study divided lymph node dissection into TLNH, PLNH, and PALNH. We found that TLNH, PLNH, and PALNH were similar for the three modalities, similar to other studies [12, 18, 28, 41]. Jung et al. [26] showed that robotic surgery has a unique advantage in lymph node dissection: RS can overcome anatomical barriers when performing lymphadenectomy. The flexibility and stability of robotic surgery makes lymphadenectomy more thorough.

With regard to hospital stay, our study showed that hospital stay with RS was significantly shorter than that with LPS and LT. The reason for this finding may be because RS is more gentle, has minor damage to the internal organs, has less postoperative pain, and has a faster return to a normal diet and normal activities.

The operation time, EBL, hospital stay, and the number of lymph nodes harvested showed significant heterogeneity in the studies that we analyzed. There are many possible reasons for this finding, such as surgical skills, surgical approaches, patients' characteristics, and learning curves of the RS system. Results from the first few procedures that are performed by a surgical team are different from those undertaken when the team has gained experience.

In conclusion, RS for endometrial cancer is a safe and effective surgical practice and has revolutionized surgical practice in endometrial cancer. Large-scale application of RS still faces a series of challenges, such as a high cost, testing, maintenance costs, and surgical costs, as important reasons for restricting the development and extensive promotion of RS. We believe that as RS technology continues to improve, its application will increase.

## Figures and Tables

**Figure 1:** 

**Figure 2:** Forest plot of the OT between the RS and LPS groups.

**Figure 3:** Forest plot of the EBL between the RS and LPS groups.

**Figure 4:** Forest plot of the OT between the RS and LT groups.

**Figure 5:** Forest plot of EBL between the RS and LT groups.

**Table 1:** Characteristics of the included studies.

Study	Country	Center	Type	Time	Age (year)	BMI (kg/m^2^)	Surgeon
RS/LPS/LT							
Bell et al., 2008	USA	Single	Retrospective cohort	2000.5-2007.6	63.0 ± 10.1	33.0 ± 8.5	S
					68.4 ± 11.9	31.9 ± 9.8	
					72.3 ± 12.5	31.8 ± 7.7	
Boggess et al., 2008	USA	Single	Retrospective cohort	2005.6-2007.12	61.9 ± 10.6	32.9 ± 7.6	NS
					62 ± 10.8	29 ± 6.5	
					64 ± 12.8	34.7 ± 9.2	
Coronado et al., 2012	Spain	Single	Retrospective cohort	2003-2011.6	67.3 ± 10.2	28.7 ± 4.7	NS
					65.9 ± 11.2	27.2 ± 5.3	
					64.7 ± 11.2	29.5 ± 6.6	
Chiou et al., 2015	Taiwan	Single	Retrospective cohort	2011-2013	53.6 ± 11.1	26.0 ± 5.2	S
					51.4 ± 14.2	25.6 ± 5.6	
					53.6 ± 11.3	26.1 ± 5.7	
Corrado et al., 2015	Italy	Single	Retrospective cohort	2010.8-2013.12	64 (35-90)	28 (17-80)	S
					62 (28-86)	29 (17-59)	
					63 (38-88)	29 (20-42)	
Estape et al., 2012	USA	Multi	Retrospective cohort	2002-2009	64 ± 14.5	31.5 ± 8.3	S
					60.8 ± 13.2	30.3 ± 6.9	
					64.9 ± 12.2	33.1 ± 8.2	
Jung et al., 2010	Korea	Single	Prospective cohort	2006.5-2009.1	52.9 ± 11.9	23.4 ± 3.1	NS
					49.9 ± 10.8	25.2 ± 5.1	
					50.2 ± 8.1	24.8 ± 4.0	
Johnson et al., 2017	USA	Single	Retrospective cohort	2008.10-2012.9	63.0 ± 10.9	35.5 ± 9.48	
					62.8 ± 10.7	34.3 ± 10.7	
					62.9 ± 11.1	38.4 ± 11.0	
Manchana et al., 2015	Thailand	Single	Retrospective cohort	2011.1-2014.12	56 (48-61)	26.8 (22.7-35.6)	NR
					54 (49-62)	24.4 (21.8-28.3)	
					59 (53-65)	25.4 (22.5-30.2)	
Magrina et al., 2008	USA	Single	Prospective cohort	2004.3-2007.12	64.6 ± 11.9	30.77 ± 10.0	NR
					69.3 ± 9.4	27.32 ± 7.6	
					65.2 ± 11.4	30.5 ± 9.1	
Pulman et al., 2017	Canada	Single	Retrospective cohort	2005.1-2013.12	64.6 ± 7.3	30.8 (18.4-51.0)	NS
					63.3 ± 7.7	26 (20-40)	
					62.5 ± 11.5	32.6 (20-46.9)	
Shah et al., 2011	USA	Single	Prospective cohort	2009.1-2009.12	58.2 ± 7.57	40.5 ± 11.0	NR
					59.9 ± 10.4	29.8 ± 7.5	
					61.9 ± 9.2	35.7 ± 10.1	
RS/LPS							
CG 2010	USA	Single	Retrospective cohort	2007.12-2009.7	62 ± 8.7	32.7 ± 9.5	NS
					59.6 ± 9.75	32.32 ± 8.13	
Escobar et al., 2012	USA	Multi	Retrospective cohort	2009.4-2010.9	59.7 ± 9.2	31.4 ± 6.6	NS
					60.9 ± 12.1	31.2 ± 6.7	
Fagotti et al., 2012	Italy	Multi	Retrospective cohort	2009.2-2011.6	63 (36-85)	28 (22-25)	NR
					58 (37-84)	27 (17-46)	
Lim et al., 2011	USA	Single	Prospective cohort	2008.3-2010.7	62.1 ± 8.4	31 ± 8.8	S
					61.6 ± 11.8	29.9 ± 7.0	
Mäenpää et al., 2016	Finland	Single	RCT	2010.11-2013.10	67 (43-84)	29 (20-46)	NS
					70 (48-83)	29 (20-45)	
Seror et al., 2014	France	Single	Retrospective cohort	2002.1-2011.12	66.3 ± 2.9	24.95 ± 1.35	NS
					66.9 ± 2.3	25.35 ± 0.95	
Seamon et al., 2009	USA	Single	Prospective cohort	2006.1-2008.4	59 ± 8.9	34.3 ± 9	S
					57 ± 11	28.7 ± 6.9	
Turunen et al., 2013	Finland	Single	Retrospective cohort	2009.5-2013.1	65.4 ± 8.5	28.2 ± 5.7	S
					67.4 ± 10.6	28.8 ± 5.9	
Venkat et al., 2012	USA	Single	Retrospective cohort	2008-2010			S
							
RS/LT							
DeNardis et al., 2008	USA	Single	Retrospective cohort	2006.7-2007.8	58.9 ± 10.3	28.5 ± 6.4	NR
					62.5 ± 10.8	34.0 ± 9.3	
ElSahwi et al., 2012	USA	Single	Retrospective cohort	2006.9-2010.9	62.4 ± 9.9	34.5 ± 9.2	S
					65 ± 12	33 ± 9	
Eklind et al., 2015	Sweden	Single	Prospective cohort	2010.9-2012.12	66 (47-87)	29 (19-46)	S
					66 (44-84)	29 (19-44)	
Goel et al., 2011	USA	Single	Retrospective cohort	2006.6-2008.6	59.5 ± 1.43	39.3 ± 2.03	S
					66.5 ± 1.97	32.2 ± 2.03	
Park et al., 2015	USA	Single	Retrospective cohort	2001.1-2012.7	60 (24-88)	30.7 (18.1-66.9)	NS
					60 (26-91)	30.4 (15.6-68.7)	
Mok et al., 2012	Singapore	Single	Retrospective cohort	2008.8-2010	56.2 ± 9.8	25.6 ± 5.3	NS
					53.6 ± 13.9	26.1 ± 7.2	

## Data Availability

Some or all data, models, or code generated or used during the study are available from the corresponding author by request.

## Supplementary Materials

Supplementary Materials Figure S1: forest plot of intraoperative complications between the RS and LPS groups. Figure S2: forest plot of postoperative complications between the RS and LPS groups. Figure S3: forest plot of blood transfusion between the RS and LPS groups. Figure S4: forest plot of conversion between the RS and LPS groups. Figure S5: forest plot of TLNH between the RS and LPS groups. Figure S6: forest plot of the number of PLNH between the RS and LPS groups. Figure S7: forest plot of the number of PALNH between the RS and LPS groups. Figure S8: forest plot of hospital stay between the RS and LPS groups. Figure S9: forest plot of intraoperative complications between the RS and LT groups. Figure S10: forest plot of postoperative complications between the RS and LT groups. Figure S11: forest plot of blood transfusion between the RS and LT groups. Figure S12: forest plot of TLNH between the RS and LT groups. Figure S13: forest plot of the number of PLNH between the RS and LT groups. Figure S14: forest plot of the number of PALNH between the RS and LT groups. Figure S15: forest plot of hospital stay between the RS and LT groups. Figure S16: (a) funnel plots for intraoperative complications of RS vs. LPS; (b) funnel plots for intraoperative complications of RS vs. LT. Figure S17: MOOSE checklist. Table S1: NOS score of the study.
